# Exosomal CXCL14 Contributes to M2 Macrophage Polarization through NF-*κ*B Signaling in Prostate Cancer

**DOI:** 10.1155/2022/7616696

**Published:** 2022-05-27

**Authors:** Hong-Yang Tian, Qi Liang, Zhen Shi, Hang Zhao

**Affiliations:** ^1^Department of Urology, The First Affiliated Hospital of Jinzhou Medical University, Jinzhou, China; ^2^Department of Urology Surgery, Dalinghe Hospital Affiliated to Medical College of Jinzhou Medical University, Jinzhou 121206, China; ^3^Department of Hepatobiliary Diseases, The First Affiliated Hospital of Jinzhou Medical University, Jinzhou, China

## Abstract

Chemokine (C-X-C motif) ligand 14 (CXCL14) plays a critical role in maintaining homeostasis and inflammation in the local cell environment and regulating cancer progression. However, the role of CXCL14 in prostate cancer (PC) has not been fully investigated. In this study, the expression of CXCL14 was determined in PC tumor tissues by qRT-PCR and immunohistochemistry assay. Wound healing, invasion, colony formation, cell proliferation, and apoptosis assays were performed to evaluate the role of CXCL14 in PC progression. Exosomes were isolated from PC cell-condition medium by using ultracentrifugation assay and identified by using transmission electron microscopy and nanoparticle tracking analysis. M2 macrophage polarization-associated genes were measured by using qRT-PCR and Western blot assays. A PC xenograft mouse model was used to assess the role of CXCL14 in tumor growth in vivo. The results showed that CXCL14 was significantly upregulated in PC tissues and was positively correlated with pathological stages, lymph node metastasis, and angiolymphatic invasion. The positive correlations were also observed between CXCL14 and PD-L1 and IL-10. Knockdown CXCL14 dramatically inhibited PC cell proliferation, invasion, and colony formation, but not apoptosis. CXCL14 promoted M2 macrophage polarization through the NF-*κ*B signaling pathway and exosome-mediated mechanism. Moreover, CXCL14 knockdown inhibited tumor growth in vivo. Taken together, exosomal CXCL14 promoted M2 macrophage polarization through the NF-*κ*B signaling pathway and contributed to PC progression.

## 1. Introduction

Prostate cancer (PC) has emerged as the fifth leading cause of cancer-associated death in men around the world and the second wild-spreading devastating tumor, after lung cancer, in males [1, 2]. According to the data from GLOBOCAN, 1,276,106 new cases of PC were documented worldwide in 2018, with a higher incidence in the Western countries [1]. In China, 120,000 new cases were reported in 2016, and PC is ranked the ninth malignant tumor in men [3, 4]. Even if the 5-year survival rate of PC is more than 99%, patients with metastatic PC only have about 31% of the 5-year survival rate [5]. Moreover, PC in the advanced stage is generally regarded as incurable [5]. Thus, although notable progress has been achieved in the diagnosis and treatment of PC, the comprehensive understanding of the molecular basis of PC progression remains to be elucidated.

Chemokines (chemotactic cytokines) are a group of small signaling proteins, 8-10 kDa, that are produced in almost all cell types [6]. Chemokines play a critical role in regulating directed chemotaxis of surrounding responsive cells and maintaining homeostasis and inflammation in the local extracellular environment [7]. As a relatively newly discovered member, chemokine (C-X-C motif) ligand 14 (CXCL14) is widely distributed in normal skin epithelia and is involved in immune cell maturation and recruitment [7]. Meanwhile, CXCL14 is a vital regulator in the antimicrobial and antitumoral processes [8, 9]. It has been demonstrated that CXCL14 is highly expressed in various tumors, including pancreatic cancer [10], lung cancer [11], and colorectal cancer [12]. For PC, the upregulation of CXCL14 is reported in localized PC and is positively correlated with PC progression [13]. Cancer-associated fibroblasts- (CAFs-) derived CXCL14 functions as a stimulator to promote PC development and tumor growth [14].

Macrophages are critical factors for establishing a protumor inflammatory microenvironment associated with tumor cell proliferation, migration, invasion, and angiogenesis [15]. In general, tumor-associated macrophages (TAMs) display two distinct polarized forms: classical (M1) form characterized by enhancing immune responses and acting as antitumor factors and alternative (M2) form characterized by suppressing immune activities and promoting tumorigenesis [16]. As multifunctional regulators, M2 macrophages secrete a high level of programmed death-ligand 1 (PD-L1) to induce checkpoint blockade of T cells, thereby promoting immunosuppressive responses to tumor cells [17]. Meanwhile, M2 macrophages produce interleukin-10 (IL-10), an immunosuppressive cytokine, to suppress antitumor immune responses [18]. Thus, the molecular and cellular interplay between macrophage M1 and M2 forms appear to be essential for determining cancer progression. However, the effect of CXCL14 in M2 macrophage polarization has not been investigated in PC. Thus, this study is aimed at determining the role of CXCL14 in PC progression, especially M2 macrophage polarization.

## 2. Materials and Methods

### 2.1. Ethics Statement

All human sample procedures and experimental protocols were approved by the Ethics Committee of the First Affiliated Hospital of Jinzhou Medical University, and the methods were carried out in accordance with the Declaration of Helsinki [19]. Informed consent was obtained from each patient. All animal experiments protocols were approved by the Institutional Animal Care and Use Committee of the First Affiliated Hospital of Jinzhou Medical University and were carried out in accordance with the recommendations in the Guide for the Care and Use of Laboratory Animals of the National Institutes of Health.

### 2.2. Patient Samples

PC tumor tissues and paired adjacent normal tissues (*n* = 28) were obtained from 28 patients who underwent surgical resection from February 2016 to February 2017. Blood samples were collected from all PC patients and healthy individuals (*n* = 24). The diagnosis of PC was verified by histopathological evaluation and clinical examination. After resection, all samples were immediately frozen and stored in liquid nitrogen for subsequent analysis. The clinicopathological characteristics of the PC patients were summarized in Table 1.

### 2.3. Cell Culture

The human PC cell lines (LNCaP and PC-3) and human monocyte cell line THP-1 were obtained from the Institute of Biochemistry and Cell Biology of the Chinese Academy of Sciences (Shanghai, China). PC-3 and THP-1 cells were cultured in the RPMI-1640 medium (Gibco, USA). LNCaP cells were cultured in DMEM-F12 medium (Gibco, USA). All cell culture media were supplemented with 10% fetal bovine serum (FBS), 1 mg/ml streptomycin, and 100 units/ml penicillin at 37°C under 5% CO_2_ incubator. THP-1 cells were used to establish M0, M1, and M2 macrophages as previously described [20]. Cells were cultured for 2-3 passages and used for experiments.

### 2.4. Measurement of Plasma CXCL14

The abundance of plasma CXCL14 was measured by using Human CXCL14 ELISA kit (RayBiotech, USA). The optical density values were measured using a microplate reader at 450 nm.

### 2.5. Immunohistochemistry

Immunohistochemistry assay was performed in human or mouse PC tumor tissues as previously described [21]. Briefly, tissues were sectioned into 4 *μ*m thick sections from formalin-fixed and paraffin-embedded forms. After dewaxing, sections were incubated in 3% H_2_O_2_ solution for 30 min at room temperature to block endogenous peroxidase activities. Then, sections were microwaved for antigen retrieval in a citrate buffer. Sections were then incubated with primary antibodies CXCL14 (1 : 100), PD-L1 (1 : 100), and IL-10 (1 : 50) (Cell Signaling Technology, USA) at 4°C overnight. Slides were coverslipped after sample counterstaining. Five random regions in each section were selected to analyze under an inverted microscope. The cell images were analyzed by Image-Pro Plus 6 software (Media Cybernetics, USA).

### 2.6. Western Blot

Total protein was isolated from cells or exosomes using RIPA lysis buffer with a proteinase inhibitor. The concentration of protein was determined by Bradford Protein Assay (Bod-Rad, USA). A total of 25 *μ*g of protein along with 2 × SDS loading buffer were loaded and were separated by 12% SDS-PAGE electrophoresis and transferred electrically to PVDF membranes (Thermo Fisher Scientific, USA). Then, the membranes were blocked with 5% skim milk in PBS-0.05% Tween 20 for 2 h at room temperature. The primary antibodies for GADPH, CXCL14, PD-L1, CD81, Hsp70, and NF-*κ*B (Santa Cruz Biotechnology, USA) were used to incubate with membranes overnight at 4°C. Then, membranes were incubated with corresponding secondary antibodies for 1 h at 37°C and visualized by enhanced chemiluminescence assays (Thermo Fisher Scientific, USA). The optical density of protein bands was quantified by using ImageJ software.

### 2.7. Quantitative Real-Time PCR

Total RNA was isolated from tissues or cells using TRIzol reagent (Thermo Fisher Scientific, USA). Reverse transcription was performed using M-MLV Reverse Transcriptase (RNase H) kit (GeneCopoeia, USA). Quantitative real-time PCR was carried out on the ABI7900 system (Applied Biosystems by Life Technologies, USA) using Power SYBR Green (Takara, Japan) according to the manufacturer's instructions. Raw PCR data were analyzed using the *ΔΔ*CT method [22]. *β*-Actin was used as the reference gene. The primer information was as follows: *β*-actin: forward 5′-ACTGGAACGGTGAAGGTGA C-3′, reverse 5′-AGAGAAGTGGGGTGGCTTTT-3′; CXCL14: forward 5′-TCCGGTCAGCATGAGGCTCC-3′, reverse 5′- CACCCTATTCTTCGTAGACC-3′; CD206: forward 5′-CTCTGTTCAGCTATTGGACGC-3′, reverse 5′- CGGAATTTCTGGGATTCAGCTTC-3′; IL-10: forward 5′-GAGATGCCTTCAGCAGAGTGAAGA-3′, reverse 5′- AGGCTTGGCAACCCAGGTAAC-3′; CD64: forward 5′-CTTCTCCTTCTATGTGGGCAGT-3′, reverse 5′-GCTACCTCGCACCAGTATGAT-3′; TNF-*α*: forward 5′-GACAAGCCTGTAGCCCATGTTGTA-3′, reverse 5′- CAGCCTTGGCCCTTGAAGA-3′; I*κ*B*α*: forward 5′-GATGGCCTCAAGAAGGAGCGCT-3′, reverse 5′- AGTGGAGATGCTGGGGTGTGCA-3′; and NF-*κ*B: forward 5′-ATGGACGATCTGTTTCCCCT-3′, reverse 5′- CGGTTTACTCGGCAGATCTT-3′.

### 2.8. Exosome Isolation

LNCaP cells were cultured in DMEM with 10% exosome-free FBS (Gibco, USA). The conditioned medium was collected after 48 h and used for exosome isolation using the ultracentrifugation assay as previously described [23]. Exosomal protein was determined by Bradford Protein Assay (Bod-Rad, USA). Exosome morphology was determined by using transmission electron microscopy (TEM). Exosome size was quantified by using nanoparticle tracking analysis (NTA) (Malvern Panalytical, UK). The expressions of exosomal markers CD81 and HSP70 were determined by Western blot.

### 2.9. Oligonucleotide Transfections

Small interfering RNAs against CXCL14 (si-CXCL14) and a random negative siRNA (si-NC) were synthesized by RiboBio Co. (Guangzhou, China). The sequences information was as follows: si-CXCL14: 5′- UGAAGAAGCUGGAAAUGAA dTdT-3′ (sense), and 3′-dTdTACUUCUUCGACCUUUACUU-5′ (antisense). Transfections of siRNAs were performed using Lipofectamine 2000 (Invitrogen, USA) according to the manufacturer's instructions. The cells were collected after 48 hours for subsequent experiments.

### 2.10. Wound Healing, Invasion, and Colony Formation Assays

Cultrex® Cell Invasion Assay Kit (R&D Systems) was used for invasion assays according to the manufacturer's protocol. Briefly, 48 hours after transfection, 1 × 10^5^ cells were counted and seeded on Matrigel inserts in serum-free medium for 20 h. Then, cells were removed from the top of the inserts, and invasive cells were fixed and stained in the polycarbonate basement membrane. For colony formation assay, 1,000 cells were seeded at the medium and allowed to grow until colonies were visible. Colonies were stained with Giemsa. For wound healing assay, when cells were confluent, 1 ml pipette tips were applied to create a homogeneous scratch wound on the monolayer. Cells were photographed at 0 and 48 h after creating the scratch. The width of scratches was quantified at three different positions (bottom, middle, and top), and the mean of width was calculated.

### 2.11. Cell Proliferation Assay

A CCK-8 assay kit was used to analyze cell proliferation (Dojindo, Japan). After siRNA transfection for 48 hours, 4,000 cells per well were seeded in 96-well plates with 200 *μ*l of culture medium. After each day of culture (total 7 days), the cells were treated with 10 *μ*l of CCK-8 solution and then incubated for 4 h at 37°C. Cell proliferation was assessed by measuring absorbance at 450 nm.

### 2.12. Apoptosis Assay

Flow cytometry analysis for apoptosis was performed 48 hours after transfection by using Annexin V-FITC/7-AAD Kit according to the manufacturer's protocol (Beckman Coulter. USA). Stained cells were evaluated by using a flow cytometer (Beckman Coulter, USA).

### 2.13. Immunofluorescence Assay

Exosomes were resuspended in PBA and stained with red PKH26 dye using a PKH26 fluorescent kit according to the manufacturer's protocol (Sigma, USA). Then, stained exosomes were incubated with PMA-pretreated THP-1 cells overnight. For subcellular location of CXCL14, anti-CXCL14 antibody (Abcam, USA) was used to incubatd with LNCaP cells. Cells were photographed by using a fluorescence microscope.

### 2.14. In Vivo Animal Experiment

C57BL/6 male mice (6 weeks) were obtained from the Chinese Academy of Sciences (Shanghai, China) and were housed in the pathogen-free animal facility with a 12 h dark-light cycle. 5 × 10^5^ exponentially growing LNCaP cells were injected subcutaneously in the right flank of each mouse (*n* = 5). When the volume of solid tumors reached 100-150 mm^3^, 5 *μ*g si-NC or si-CXCL14 was mixed with 5 *μ*l transfection reagent and was injected intratumorally into the tumor mass every 3 days for 3 weeks. Then, mice were sacrificed. Measurements were performed using a caliper, and tumor volume (mm^3^) was calculated using the formula: (length × width2)/2.

### 2.15. Statistical Analysis

All experiments were carried out in at least triplicate. Data were presented as mean ± standard deviation (SD). SPSS (18.0 version) was used for statistical analysis. Student's *t*-test was used for statistical analysis of data. Differences in clinicopathological features between groups were analyzed by chi-square tests. Correlation analysis was performed using Pearson's correlation analysis. Statistical differences were defined as follows: ^∗^*p* < 0.05, ^∗∗^*p* < 0.01, and ^∗∗∗^*p* < 0.001.

## 3. Results

### 3.1. CXCL14 Was Highly Expressed in PC Tumor Tissues

By collecting 28 pairs of PC tumor tissues and adjacent benign tissues, we first detected the mRNA abundance of CXCL14. The results showed that mRNA CXCL14 was highly upregulated in PC tissues compared with adjacent normal tissues (Figure 1(a)). The increase of CXCL14 was verified by applying the IHC assay (Figure 1(b)). The plasma level of CXCL14 was higher in PC patients relative to the healthy individuals (Figure 1(c)). Immunofluorescence assay demonstrated that CXCL14 was primarily distributed in the cellular cytoplasm and membrane, and a small amount of CXCL14 was also detected in the nucleus (Figure 1(d)). Also, the expression of CXCL14 was highly correlated with pathological stages, lymph node metastasis, and angiolymphatic invasion of patients with PC (Table 1). To investigate the role of CXCL14 in M2 macrophage polarization, the protein expressions of PD-L1 and IL-10 were measured in PC tumor tissues with high (≥50%) or low (<50%). We found that the levels of PD-L1 and IL-10 were higher in tissues with high CXCL14 expression compared with those with low CXCL14 expression (Figure 1(e)). Pearson's correlation analysis revealed that the level of CXCL14 was positively correlated with the expressions of PD-L1 and IL-10, respectively (Figures 1(f) and 1(g)). As such, these data suggest that the upregulation of CXCL14 in PC is associated with M2 macrophage polarization.

### 3.2. CXCL14 Knockdown Inhibited PC Cell Progression

To determine the role of CXCL14 in PC cells, we applied siRNA to knockdown CXCL14 in PC LNCaP and PC-3 cells (Figures 2(a) and 2(b)). The downregulation of PD-L1 mRNA expression was also observed in PC cells with CXCL14 knockdown, further verifying the positive correlation between CXCL14 and PD-L1 (Figure 2(a)). In the CCK-8 assay, PC cells treated with siRNA showed a lower level of cell proliferation relative to cells treated with siRNA negative control (Figure 2(c)). The ability of colony formation was inhibited in PC cells with CXCL14 knockdown compared with those in the control group (Figure 2(d)). CXCL14 knockdown did not impact PC cell apoptosis, as demonstrated by flow cytometry assay (Figure 2(e)). Furthermore, CXCL14 knockdown significantly suppressed the migration and invasion of PC cells, as illustrated in wound healing assay and Transwell invasion assay, respectively (Figures 2(f) and 2(g)).

### 3.3. CXCL14 Knockdown Inhibited M2 Macrophage Polarization in PC

To further investigate the role of CXCL14 in macrophage polarization, THP-1 cells were pretreated with 100 ng/ml phorbol myristate acetate (PMA) and used as M0 macrophages. PMA-treated THP-1 cells (M0) were then cocultured with PC cells with CXCL14 knockdown in the Transwell coculture system. PMA-treated THP-1 cells were further treated with IL-4 and IL-13 and used as M2 macrophage, whereas treated with IFN-*γ* and LPS to establish M1 macrophage. The M2 macrophage marker CD206 was decreased in M0 cells treated with si-CXCL14-treated PC cells, compared with those treated with si-NC-treated PC cells (Figure 3(a)). The M2-associated gene IL-10 was downregulated in macrophages cocultured with si-CXCL14-treated PC cells than those cocultured with si-NC-treated PC cells (Figures 3(b) and 3(c)). Moreover, M1 macrophage marker CD64 and M1 cytokines TNF-*α* were increased in M0 macrophages treated with PC cells with CXCL14 knockdown relative to those cocultured with PC cells treated with si-NC (Figures 3(d) and 3(e)). Collectively, these observations suggest that CXCL14 may exert a positive role in M2 macrophage polarization in PC.

### 3.4. Exosomes Mediated the Role of CXCL14 in M2 Macrophage Polarization

In this study, we observed that coculturing M0 macrophages with PC cells promoted M2 macrophage polarization. Given the well-known essential role of exosomes in intercellular communication and cancer progression [24, 25], we thus hypothesized that exosomes might be an underlying mechanism about the role of CXCL14 in M2 macrophage polarization. Then, we isolated exosomes from the LNCaP cell culture medium. By TEM and NTA, the morphology of exosomes displayed round-shaped, 50-135 nm in diameter (Figure 4(a)). The exosomal markers CD81 and Hsp70 were highly expressed in exosomes relative to cell lysis (Figure 4(b)). These data collectively suggest that exosomes were successfully isolated. Furthermore, we uncovered that the level of CXCL14 was higher in M0 macrophage treated with exosomes compared with those treated with negative control PBS (Figure 4(c)). By performing the immunofluorescence assay, we further observed that PKH26-stained exosomes were distributed in the cytoplasm of M0 macrophages (Figure 4(d)).

### 3.5. CXCL14 Contributed to M2 Macrophage Polarization through NF-*κ*B Signaling

It has been demonstrated that NF-*κ*B signaling is a crucial regulator for macrophage function in cancer progression [26, 27]. Thus, we measured the mRNA expressions of NF-*κ*B and I*κ*B*α* in M0 macrophages treated with LNCaP cells with CXCL14 knockdown. The results illustrated that both NF-*κ*B and I*κ*B*α* were reduced in M0 macrophages treated with si-CXCL14-treated LNCaP cells relative to those treated with si-NC-treated LNCaP cells (Figures 5(a) and 5(b)). Meanwhile, the effect of LNCaP cells with CXCL14 knockdown on M0 macrophages was reversed by NF-*κ*B signaling activator betulinic acid (BA), as manifested by upregulating IL-10 but lowering TNF-*α* (Figure 5(c)). The opposite role was found in M0 macrophages treated with LNCaP cells with CXCL14 knockdown as well as JSH-23, NF-*κ*B signaling inhibitor (Figure 5(d)). Furthermore, the inhibitory effect of CXCL14 knockdown on PC cell progession was reversed by the addition of BA, as illustrated by wound healing and Transwell invasion assays (Figures 5(e) and 5(f)).

### 3.6. CXCL14 Knockdown Inhibited Tumor Growth In Vivo

In this study, LNCaP cells were injected subcutaneously into nude mice to develop solid tumors until volume reached around 100-150 mm^3^. Then, si-CXCL14 and si-NC were injected intratumorally into the tumor mass every 3 days for 3 weeks. The results showed that CXCL14 knockdown significantly inhibited tumor growth in xenografts mice (Figures 6(a) and 6(b)). Meanwhile, the IHC assay demonstrated that the expressions of CXCL14, PD-L1, and IL-10 were decreased in tumor tissues of mice treated with si-CXCL14 (Figure 6(c)).

## 4. Discussion

To date, due to the relatively rare understanding of the molecular mechanism underlying PC progression, the prognosis of PC patients is still unsatisfying [28, 29]. Thus, elucidating the mechanism of PC tumorigenesis would be the urgent need for developing effective diagnostic approaches and therapies for PC patients. In this study, we reported that CXCL14 was highly expressed in PC tumor tissues and positively correlated with expressions of PD-L1 and IL-10, as well as pathological stages. We also demonstrated that CXCL14 knockdown inhibited PC cell proliferation, colony formation, invasion, and migration. More importantly, this study revealed that CXCL14 promoted M2 macrophage polarization through exosome-mediated intercellular communication by activating NF-*κ*B signaling.

As a chemokine family member, CXCL14 plays a critical role in the maturation of dendritic cells, upregulation of major histocompatibility complex- (MHC-) I, immune cell infiltration, and cell mobilization [30]. The aberrant expression profile of CXCL14 has also been reported in several cancers [31–34]. In this study, we found that CXCL14 was highly expressed in PC tumor tissues, which is agreed with several previous reports [13, 14]. Moreover, the upregulation of CXCL14 in PC was identified to be positively correlated with several clinicopathological features, including pathological stages, lymph node metastasis, and angiolymphatic invasion, suggesting that CXCL14 may serve as a potential prognostic marker for PC. Furthermore, the oncogenic role of CXCL14 was also uncovered in PC, as ministered by inhibiting PC cell progression induced by CXCL14 knockdown. As an important chemokine, the role of CXCL14 displays a cancer-type-dependent pattern, including either oncogenic or antitumor roles [7]. The possible explanation for such conflicting role of CXCL14 in cancer is associated with the origin of CXCL14: epithelial-derived CXCL14 is an antitumor factor, whereas fibroblast-derived CXCL14 is an oncogenic regulator [30]. Thus, CXCL14-based diagnosis or treatment should be applied with caution with further mechanistic studies.

In the present study, the upregulation of CXCL14 was found to be tightly correlated with the expressions of two M2 macrophage-associated factors PD-L1 and IL-10, suggesting the potential role of CXCL14 in regulating M2 macrophage polarization. It has been well-illustrated that TAMs-released PD-L1 can contribute to the immunosuppression in the tumor microenvironment by inducing macrophage polarization towards an M2-like phenotype [35]. Meanwhile, M2-polarized macrophages promote tumor progression, such as epithelial-mesenchymal transition, through IL-10 signaling pathway [36–38]. Given that PD-L1 and IL-10 are essential for the role of M2 macrophages in tumor progression and their positive correlation with CXCL14, we further demonstrated that M2 macrophage markers CD206 and IL-10 were decreased, whereas M1 macrophage markers CD64 and M1 cytokines TNF-*α* were increased in M0 macrophages with CXCL14 knockdown. These observations together suggest that CXCL14 contributes to macrophage polarization towards an M2-like phenotype. In this study, the data indicated that NF-*κ*B signaling participated in the role of CXCL14 in M2 macrophage polarization and PC progression. NF-*κ*B has been demonstrated as a critical regulator of macrophage function in tumor progression [26, 39]. Thus, the CXCL14/NF-*κ*B signaling pathway might be a potential target of anticancer therapy for PC.

Exosomes, 30 to 150 nm in diameter, are 30 to 150 nm nanosized extracellular vesicles that are released from a variety of cell types [40]. Exosomes play a critical role in intercellular communication by shuttling biofunctional molecules, including noncoding RNAs, enzymes, lipids, and DNAs, from releasing cells to recipient cells [41]. Numerous studies have demonstrated that exosomes and exosomal cargos are essential for promoting cancer progression, including M2 macrophage polarization [42, 43]. Exosomes derived from lung cancer cells promote M0 macrophages to polarize to M2 phenotype, along with changing oxygen consumption and altering the bioenergetic state [42]. Moreover, exosomes released from hypoxia-treated tumor cells facilitate M2 macrophage polarization in infiltrating myeloid cells through the microRNA let-7a and Akt-mTOR signaling pathway [44]. In this study, we reported that exosomes derived from PC LNCaP were taken up by M0 macrophages and enhanced the level of CXCL14 of the recipient macrophages. These findings suggest that exosomes mediated the role of CXCL14 in M2 macrophage polarization.

## 5. Conclusion

In conclusion, the upregulation of CXCL14 functioned oncogenic roles in PC. Exosomal CXCL14 promoted M2 macrophage polarization through NF-*κ*B signaling pathway. The findings of this study provide a novel understanding of molecular mechanisms underlying PC progression.

## Figures and Tables

**Figure 1:** CXCL14 was highly expressed in PC tumor tissues. (a) The mRNA expression of CXCL14 in 28 pairs of PC tumor tissues and adjacent benign tissues (control). (b) The protein expression of CXCL14 in PC tumor tissues and adjacent benign tissues. The data were obtained from the immunohistochemistry assay. Scale bar: 20 *μ*m. (c) The plasma level of CXCL14 in PC patients and healthy individuals, as detected by ELISA assay. (d) Subcellular localization of CXCL14. Scale bar: 25 *μ*m. (e) The protein expressions of PD-L1 and IL-10 in PC tissue with high CXCL14 expression (≥50%) or low CXCL14 expression (<50%). The data were obtained from the immunohistochemistry assay. Scale bar: 20 *μ*m. (f) Pearson correlation analysis for the expressions of CXCL14 and PD-L1. (g) Pearson correlation analysis for the expressions of CXCL14 and IL-10. ^∗^*p* < 0.05, ^∗∗^*p* < 0.01, and ^∗∗∗^*p* < 0.001.

**Figure 2:** CXCL14 knockdown inhibited PC cell progression. (a) The mRNA expressions of CXCL14 and PD-L1 in PC LNCaP and PC-3 cells treated with siRNA against CXCL14 (si-CXCL14) or siRNA negative control (si-NC). (b) The protein expressions of CXCL14 and PD-L1 in PC LNCaP and PC-3 cells treated with siRNA against CXCL14 (si-CXCL14) or siRNA negative control (si-NC). (c) CCK-8 assay for LNCaP and PC-3 cells treated with si-NC or si-CXCL14. (d) Colony formation assay for LNCaP and PC-3 cells treated with si-NC or si-CXCL14. (e) Flow cytometry analysis for LNCaP and PC-3 cells treated with si-NC or si-CXCL14. (f) Wound healing assay for LNCaP and PC-3 cells treated with si-NC or si-CXCL14. (g) Transwell invasion assay for LNCaP and PC-3 cells treated with si-NC or si-CXCL14. Scale bar: 25 *μ*m; ^∗^*p* < 0.05, ^∗∗^*p* < 0.01, and ^∗∗∗^*p* < 0.001.

**Figure 3:** CXCL14 knockdown inhibited M2 macrophage polarization in PC. (a) The mRNA expression of M2 macrophage marker CD206 in PMA-pretreated THP-1 cells (M0), IL-4- and IL-13-treated M0 cells (M2), and M0 cells treated with PC cells with or without CXCL14 knockdown. (b) The mRNA expression of M2 macrophage-associated gene IL-10 in M0, M2, and M0 macrophage treated with PC cells with or without CXCL14 knockdown. (c) Immunofluorescence assay for the mRNA expression of M2 macrophage-associated gene IL-10 in M0, M2, and M0 macrophage treated with PC cells with or without CXCL14 knockdown. Scale bar: 25 *μ*m. (d) The mRNA expression of M1 macrophage marker CD64 in PMA-pretreated THP-1 cells (M0), IFN-*γ*- and LPS-treated M0 cells (M1), and M0 cells treated with PC cells with or without CXCL14 knockdown. (e) The mRNA expression of M1 cytokines TNF-*α* in M0, M1, and M0 cells treated with PC cells with or without CXCL14 knockdown. ^∗^*p* < 0.05, ^∗∗^*p* < 0.01, and ^∗∗∗^*p* < 0.001.

**Figure 4:** Exosomes mediated the role of CXCL14 in M2 macrophage polarization. (a) Transmission electron microscopy (TEM) and nanoparticle tracking analysis (NTA) for the morphology and size of exosomes derived from LNCaP cells. Scale bar: 100 *μ*m. (b) The protein expressions of exosomal markers CD81 and Hsp70 in LNCaP cell lysis or exosomes derived from LNCaP cells. (c) The protein expression of CXCL14 in PMA-pretreated THP-1 cells (M0) treated with PBS (NC) or exosomes derived from LNCaP cells. (d) Immunofluorescence assay for PMA-pretreated THP-1 cells (M0) treated with exosomes (red) derived from LNCaP cells. Scale bar: 25 *μ*m. ^∗^*p* < 0.05, ^∗∗^*p* < 0.01, and ^∗∗∗^*p* < 0.001.

**Figure 5:** CXCL14 contributed to M2 macrophage polarization through NF-*κ*B signaling. (a) The mRNA expressions of I*κ*B*α* and NF-*κ*B in PMA-pretreated THP-1 cells (M0) coculturing with LNCaP cells with or without CXCL14 knockdown. (b) The protein expression of NF-*κ*B in M0 macrophages coculturing with LNCaP cells with or without CXCL14 knockdown. (c) The mRNA expressions of IL-10 and TNF-*α* in M0 macrophages treated with LNCaP cells without CXCL14 knockdown, LNCaP cells with CXCL14 knockdown, or LNCaP cells with CXCL14 knockdown plus NF-*κ*B signaling activator betulinic acid (BA). (d) The mRNA expressions of IL-10 and TNF-*α* in M0 macrophages treated with LNCaP cells without CXCL14 knockdown, LNCaP cells with CXCL14 knockdown, or LNCaP cells with CXCL14 knockdown plus NF-*κ*B signaling inhibitor JSH-23. (e) Wound healing assay for LNCaP cells treated with si-NC, si-CXCL14, or si-CXCL14 plus BA. Scale bar: 25 *μ*m. (f) Transwell invasion assay for LNCaP and PC-3 cells treated with si-NC, si-CXCL14, or si-CXCL14 plus BA. ^∗^*p* < 0.05, ^∗∗^*p* < 0.01, and ^∗∗∗^*p* < 0.001.

**Figure 6:** CXCL14 knockdown inhibited tumor growth in vivo. (a) Representative image of tumor tissues. (b) The volume of tumor tissues of PC xenografts mice treated with siRNA against CXCL14 (si-CXCL14) or siRNA negative control (si-NC). (c) The protein expressions of CXCL14, PD-L1, and IL-10 in tumor tissues of xenografts mice treated with si-CXCL14 or si-NC. ^∗^*p* < 0.05, ^∗∗^*p* < 0.01, and ^∗∗∗^*p* < 0.001.

**Table 1:** Clinicopathological features of PC patients and their relationship with CXCL14 expression.

Characteristics	Cases (%) (*n* = 28)	CXCL14 expression (%)		*p* value
		Higher (≥50%)	Lower (<50%)	
*Age*				
<65	13 (46%)	6 (46%)	7 (54%)	0.138
≥65	15 (54%)	8 (53%)	7 (47%)	
*Pathological stage*				
T1	11 (39%)	7 (64%)	4 (36%)	0.007
T2/T3	17 (61%)	14 (82%)	3 (18%)	
*Lymph node metastasis*				
Negative	13 (46%)	8 (62%)	5 (38%)	0.012
Positive	15 (54%)	11 (73%)	4 (27%)	
*Angiolymphatic invasion*				
Negative	16 (57%)	9 (56%)	7 (44%)	0.028
Positive	12 (43%)	8 (67%)	4 (33%)	
*Preoperative PSA*				
<4 ng/ml	16 (57%)	9 (56%)	7 (44%)	0.126
≥4 ng/ml	12 (42%)	7 (58%)	5 (42%)	
*Gleason score*				
<8	12 (43%)	7 (58%)	9 (42%)	0.281
≥8	16 (57%)	6 (38%)	6 (62%)	

## Data Availability

The datasets used during the present study are available from the corresponding author upon reasonable request.
